# Construction of Standard Fast Medical Procedures for Traumatic Shock and Its Application Effects

**DOI:** 10.1155/2022/2055925

**Published:** 2022-10-11

**Authors:** Yan Wang, Siqi Luo

**Affiliations:** The Nanhua Affiliated Hospital, Department of Operating Room, Hengyang Medical School, University of South China, Hengyang 421001, Hunan, China

## Abstract

**Objective:**

To explore the construction of standard fast medical procedures for traumatic shock and its application effects.

**Methods:**

84 patients with traumatic shock were admitted to emergency department of the hospital between January 2018 and January 2020. Using random number table method, the patients were divided into the control group (was given emergency treatment by routine emergency rescue procedures) and the study group (was given emergency treatment by standard fast medical procedures) with 42 patients in each group. The treatment time (rescue time, consultation time in each department, and examination time), shock index (SI), blood pressure fluctuation range, urine output, serum lactate (LAC) level, activated partial thromboplastin time (APTT), and international normalized ratio (INR) were recorded. The incidences of complications in the two groups within 3 days were counted.

**Results:**

The rescue time, consultation time, and examination time of the study group were shorter than those of the control group (*P* < 0.05). After 18 h of treatment, the SI, blood pressure fluctuation range, LAC, and APTT in the study group were lower or shorter than those in the control group (*P* < 0.05), while urine volume and INR were higher than those in the control group (*P* < 0.05). Within 3 days of treatment, the incidence of complications in the study group was 5.41% lower than that in the control group which was 24.14% (*P* < 0.05).

**Conclusion:**

Standard fast medical procedures can effectively shorten the time of each stage of emergency treatment for traumatic shock, which allows patients to receive effective treatment in the shortest time while improving shock symptoms and reducing related complications.

## 1. Introduction

The post-traumatic body is affected by multiple factors such as tissue damage, fractures, and decreased circulating blood volume, which will cause multisystem post-traumatic reactions. When the body's circulating blood volume is insufficient and the microcirculation of multiple organs fails, it will lead to shock [1, 2]. Traumatic shock is more prone to multiple organ dysfunction syndrome (MODS) than simple hemorrhagic shock. During its pathophysiology, ischemia-reperfusion injury induces a cascade effect of cellular signalling, leading to enhanced neuroendocrine activity; activation and release of various chemical mediators, cytokines, and oxygen radicals, which can cause a nonspecific stress response; increase vascular permeability; and lead to necrosis and disintegration of damaged tissues, further reducing circulating blood volume and aggravating tissue ischemia [3, 4]. Patients with this disease not only have primary trauma but also multisystem functional damage, often severe blood loss, fluid loss, and symptoms of pain and anxiety [5]. The treatment of traumatic shock focuses on timely control of inflammation to avoid the further development and deterioration of systemic inflammatory response. The basic first aid measures include reasonable management of tissue damage, control of bleeding, volume expansion, sedation, and analgesia [6]. The standardization of emergency procedures and the timely and efficient rescue are crucial for the rescue of traumatic shock and the life of patients and should also be the focus of the construction of the medical emergency system. The purpose of this study is to explore the specific construction and clinical application effect of standard fast medical procedures for traumatic shock.

## 2. Materials and Methods

### 2.1. General Information

A total of 84 patients with traumatic shock admitted to the emergency department of our hospital from January 2018 to January 2020 were selected as the research subjects. The patients were divided into the control group and the study group by random number table method, with 42 cases in each group. The control group consisted of 24 males and 18 females; the age ranged from 18 to 66 years, with an average of (38.24 ± 6.33) years; causes of shock include the following: 16 cases of impact and abrasions; 10 cases of stab wounds, contusions, and lacerations; 8 cases of crush injuries; and 8 cases of other injuries; type of wound included the following: there were 27 open wounds and 15 closed wounds; injury sites are as follows: 8 cases of head, face, and neck; 10 cases of chest (back); 12 cases of abdomen (waist); 5 cases of limbs; 3 cases of pelvis and spine; and 4 cases of multiple injuries. The study group consisted of 28 males and 14 females; the age ranged from 18 to 64 years, with an average of (37.34 ± 6.12) years; causes of shock are as follows: 14 cases of impact and abrasions; 9 cases of stab wounds, contusions, and lacerations; 7 cases of crush injuries; and 12 cases of other injuries; type of wound includes the following: there were 30 open wounds and 12 closed wounds; injury sites are as follows: 6 cases of head, face, and neck; 10 cases of chest (back); 13 cases of abdomen (waist); 6 cases of limbs; 2 cases of pelvis and spine; and 5 cases of multiple injuries. There was no significant difference in general data between the two groups (*P* > 0.05), which was comparable. This study met ethical standards.

### 2.2. Inclusion Criteria

Inclusion criteria are as follows:(1) should have a clear history of trauma, meet the surgical diagnostic criteria [7], and be diagnosed as traumatic shock; (2) trauma index (TI) > 10; (3) all patients were admitted to hospital 24 hours after trauma; (4) the patient's family members were informed of the rescue purpose, plan, and risks, and the family members agreed to the treatment.

### 2.3. Exclusion Criteria

Exclusion criteria are as follows:(1) those who died before hospital or were transferred midway; (2) those who had serious medical diseases; (3) those who gave up treatment.

### 2.4. Nursing Methods

The control group adopted the routine emergency rescue procedures: prehospital first aid and in-hospital first aid, treatment of primary injury, effective control of active bleeding, cardiopulmonary resuscitation, keep the patient's airway unobstructed and establish venous access, replenish body fluids, closely monitor vital signs and blood oxygen saturation, etc., cooperate with doctors to actively rescue, observe the patient's condition changes, send information to doctors in a timely manner, confirm valid medical orders, and implement them.

The study group adopted standard fast medical procedures: ① set up a care support group of trauma center, formulate emergency rescue plans, divide labor among members, clarify functions, and the team leader is responsible for coordinating the emergency process such as personnel scheduling to ensure the orderly progress of the emergency process; ② in the prehospital emergency, check and evaluate the patient's trauma, shock degree, and vital signs; check whether the patient has active bleeding or hidden injury; and classify the patient according to the degree of injury; hemostasis, opening of venous access, and keeping the airway open, etc. Basic first aid measures, and dynamic monitoring of patients' vital signs; after preliminary assessment and judgment, the information is fed back to the emergency room and related departments in the hospital, so that information can be effectively communicated, so as to formulate treatment plans, clarify the division of medical care, coordinate staff in various departments, and prepare rescue drugs and equipment; ③ quickly enter the EICU through the green channel and briefly report the patient's injury, and the in-hospital care support group of trauma center will quickly make a judgment on the patient's condition, carry out in-hospital first aid, stabilize the patient's vital signs (focus on blood pressure, breathing, heart rate, and consciousness), and control activities; tracheal intubation or incision can be done to establish 2-3 circulation paths if necessary; for changes in vital signs, perform cardiopulmonary resuscitation, antishock, fluid resuscitation (crystalloid followed by colloid, low-pressure resuscitation, and hemostatic resuscitation), hemostasis, pain relief, and oxygen inhalation; inquire about the patient's trauma history in detail and perform a careful physical examination. After the attending physician prescribes the relevant biochemical examination and auxiliary imaging examination, the nurse will review and notify the relevant examination department, who will be escorted to the examination department by a special person to complete the examination, and invite multiple departments for consultation; give patients deterministic treatment, such as timely hemostasis, debridement, bandaging, and other treatments for trauma patients, and patients with rib fractures and thoracic injuries, pay attention to whether the patient has hemothorax, pneumothorax, etc., and can be given thoracic-closed drainage treatment according to the actual condition; ④ for patients who need surgery, timely feedback the patient's condition to the operating room. The EICU is ready for blood preparation. After the blood pressure is stabilized, the emergency doctor and the responsible nurse are quickly escorted to the operating room, and the preoperative preparations are handed over. After the vital signs are stabilized out of the room, do a seamless handover; ⑤ during the rescue process, it is also necessary to actively communicate with the patient's family member, inform the patient's condition change, and comfort the family member.

### 2.5. Observation Indicators

Observation indicators are as follows: (1) treatment time: record the rescue time after admission, the consultation time of each department (the time from admission to the consultation opinion), and the examination time (the time required to complete the main biochemical and imaging examinations); (2) record the shock index (SI), blood pressure fluctuation range, and urine output of the patient after 18 hours of treatment, among them, SI = pulse rate/systolic blood pressure, SI < 0.5 means no shock, 1.0 < SI < 1.5 indicates shock, and SI > 2.0 indicates severe shock; (3) serum lactate (LAC) level, activated partial thromboplastin time (APTT), and international normalized ratio (INR): venous blood was collected from patients before and 18 hours after treatment; (4) the incidence of complications [disseminated intravascular coagulation (DIC), MODS, acute respiratory distress syndrome (ARDS), and infection] within 3 days of treatment.

### 2.6. Statistical Methods

SPSS 20.0 statistical software was used for data analysis. The enumeration data was represented by *n* (%), and the *χ*^2^ test was performed; the measurement data was represented by ($\bar{x}\pm s$), and the *t*-test was performed, the test level was *α* = 0.05, and *P* < 0.05 was statistically significant.

## 3. Results

### 3.1. Treatment Time

The rescue time, consultation time, and examination time in the study group were shorter than those in the control group (*P* < 0.05), as shown in Table 1.

After 18 hours of treatment, the SI and blood pressure fluctuation range in the study group were smaller than those in the control group (*P* < 0.05), but the urine output was more than that in the control group (*P* < 0.05), as shown in Table 2.

### 3.2. LAC, APTT, and INR Levels

After 18 hours of treatment, the LAC and APTT of the study group were lower than those of the control group (*P* < 0.05), and the INR was higher than that of the control group (*P* < 0.05), as shown in Table 3.

### 3.3. Complications

Within 3 days of treatment, the incidence of complications in the study group was 5.41% lower than that in the control group 24.14% (*P* < 0.05), as shown in Table 4.

## 4. Discussions

Traumatic shock is a common surgical emergency, which often leads to damage to the patient's body organs, severe instability of vital signs, and rapid disease progression, which is prone to extreme deterioration and death [8]. Therefore, timely and effective treatment is of great significance to save the lives of patients. In patients with acute trauma, the injury should be quickly assessed, early shock symptoms should be identified, primary trauma should be prioritized, and emergency symptoms such as active bleeding and airway obstruction should be dealt with [9].

Patients with trauma need to be treated as effectively as possible in the shortest possible time after their injury. In emergency, medical staff also needs to cooperate closely, evaluate and judge the patient's condition, and take targeted treatment measures to improve the patient's symptoms in the shortest time [10]. This study is to explore the specific construction and clinical application effect of standard fast medical procedures for traumatic shock. The results of this study showed that the rescue time, consultation time, and examination time of the study group were shorter than those of the control group, and the intervention was also higher than that of the control group, suggesting that standard fast medical procedures can effectively shorten the treatment time, improve treatment efficiency, and improve patient safety. Analyze the causes: the establishment of a first aid team led by a team leader allows for a clear division of labour within the team and the development of a scientific first aid plan following evidence-based principles. The establishment of emergency rescue plans can avoid panic and blindness in the rescue process and is also conducive to efficient handling of emergencies, improving the effectiveness of rescue and avoiding the waste of personnel and resources. Prehospital trauma and shock assessment, which classifies patients according to their injuries, can be effective in improving the efficiency of treatment, ensuring that critically ill patients receive priority treatment and avoiding confusion in emergency situations. Also, the implementation of the standard fast medical procedures is patient-centered, by carrying out information linkage between multiple departments, they can communicate and discuss the patient's situation in a timely manner, clearly divide the work, cooperate with each other, do their own work in an orderly manner, then develop the best treatment plan for the patient, and ensure good treatment equipment conditions, so that the patient's treatment process is systematic and continuous, thus ensuring the success rate of patient treatment [11, 12]. The green channel approach can make up for the defects of the traditional emergency route, remove the prehospital obstacles as much as possible, and ensure that the patients are quickly admitted to the emergency room and receive treatment in the shortest time, and its rapidity can improve the treatment efficiency [13, 14].

Fluid resuscitation is an effective means to stabilize hemodynamics and restore the body's circulating blood volume. Patients with shock are often treated with fluid resuscitation, and changes in blood pressure fluctuations, heart rate, and urine output should be observed in real time. Coagulopathy, hypothermia, and acidosis are the “post-traumatic lethal triad,” which can be induced by massive fluid resuscitation [15]. INR and APTT are effective indicators for monitoring coagulation function and the occurrence of DIC [16], and LAC can reflect the severity of shock and hypoperfusion, as well as the level of oxygenation, and serve as indicators for judging metabolic disorders and prognosis [17]. The results of this study showed that after 18 h of treatment, the SI, blood pressure fluctuation range, LAC, and APTT in the study group were lower or shorter than those in the control group, while the urine volume and INR were higher than those in the control group, and the incidence of related complications within 3 days was lower than that of the control group, suggesting standard fast medical procedures can improve the patient's treatment efficiency, promote the improvement of the patient's shock symptoms, reduce the patient's blood pressure range, relieve the coagulation disorder, and reduce the incidence of complications. Analyze the causes: in the standard fast medical procedures, nurses cooperate with doctors to carry out resuscitation work, effectively implement effective instructions from doctors, resuscitate patients with fluids, closely observe changes in relevant index data, and use timely and effective low-pressure resuscitation and hemostatic resuscitation, which can not only ensure effective blood supply to vital organs but also improve the body's oxygen supply, reduce the fluctuation of blood pressure, avoid the damage of blood pressure fluctuations to the organs, and also correct the symptoms of shock in patients and prevent the dilution of coagulation factors and cause coagulation disorders [18].

In conclusion, the application of standard fast medical procedures in traumatic shock treatment can shorten the treatment time, improve the treatment efficiency, promote the relief of symptoms, and reduce the risk of related complications. This shows that the construction of standard fast medical procedures has high clinical value, but the construction of this research process is still insufficient, and it is still necessary to further optimize the nursing functions and division of labor management in the implementation process, as well as the rescue process and execution feasibility, so as to be more conducive to the rescue and treatment of patients.

## Figures and Tables

**Table 1:** Comparison of treatment time data between the control group and the study group (*n* = 42, $\bar{x}\pm s$, min).

Group	Rescue time	Consultation time	Examination time
Control group	36.52 ± 8.66	25.67 ± 6.25	23.87 ± 5.92

Study group	30.46 ± 8.47	21.33 ± 5.86	20.74 ± 5.73

*T*	3.242	3.283	2.462

*P*	0.002	0.002	0.016

SI, blood pressure fluctuation range, and urine output.

**Table 2:** Comparison of SI, blood pressure fluctuation range, and urine output between the control group and the study group after 18 hours of treatment ($\bar{x}\pm s$).

Group	*n*	SI	Blood pressure fluctuation range (mmHg)	Urine output (ml/h)
Control group	29	1.02 ± 0.12	27.54 ± 8.63	33.41 ± 5.11
Study group	37	0.71 ± 0.08	20.12 ± 8.34	36.52 ± 5.87
*T*		12.562	3.533	2.260
*P*		<0.001	<0.001	0.027

*Note.* Patients who died within 18 hours of admission were excluded.

**Table 3:** Comparison of LAC, APTT, and INR levels between the control group and the study group ($\bar{x}\pm s$).

Group	*n*	LAC (mmol/L)		APTT (s)		INR	
		Before treatment	18 h after treatment	Before treatment	18 h after treatment	Before treatment	18 h after treatment
Control group	29	4.96 ± 1.16	3.62 ± 0.86^*∗*^	60.35 ± 9.54	52.26 ± 8.86^*∗*^	1.21 ± 0.13	1.32 ± 0.24^*∗*^
Study group	37	4.77 ± 1.12	2.27 ± 0.77^*∗*^	61.26 ± 9.67	47.68 ± 8.71^*∗*^	1.24 ± 0.17	1.47 ± 0.31^*∗*^
*T*		0.673	6.715	0.382	2.104	0.787	2.148
*P*		0.503	<0.001	0.704	0.040	0.434	0.036

*Note.* Compared with before treatment, ^*∗*^*P* < 0.05.

**Table 4:** Comparison of the incidence of complications in the control group and the study group within 3 days of treatment (cases, %).

Group	*n*	DIC	MODS	ARDS	Infection	Total incidence
Control group	29	2	1	1	3	7 (24.14%)
Study group	37	0	0	0	2	2 (5.41%)
*χ * ^2^						4.844
*P*						0.028

## Data Availability

The raw data supporting the conclusion of this article will be available by the authors without undue reservation.

## References

[1] Cole E., Gillespie S., Vulliamy P., Brohi K., Organ D. (2020). Trauma (ORDIT) study collaborators. “Multiple organ dysfunction after trauma”. *British Journal of Surgery*.

[2] Ziesmann M. T., Marshall J. C. (2018). Multiple organ dysfunction: the defining syndrome of sepsis. *Surgical Infections*.

[3] Jones A. R., Miller J. L., Jansen J. O., Wang H. E. (2021). Whole blood for resuscitation of traumatic hemorrhagic shock in adults. *Advanced Emergency Nursing Journal*.

[4] Kuo K., Palmer L. (2022). Pathophysiology of hemorrhagic shock. *Journal of Veterinary Emergency and Critical Care*.

[5] Li Y., Zhang L. M., Zhang D. X. (2020). CORM-3 ameliorates neurodegeneration in the amygdala and improves depression- and anxiety-like behavior in a rat model of combined traumatic brain injury and hemorrhagic shock. *Neurochemistry International*.

[6] Eastridge B. J., Holcomb J. B., Shackelford S. (2019). Outcomes of traumatic hemorrhagic shock and the epidemiology of preventable death from injury. *Transfusion*.

[7] Hardcastle T. C., Steyn E., Boffard K. (2011). Guideline for the assessment of trauma centres for South Africa. *South African Medical Journal*.

[8] Ma X., Aravind A., Pfister B. J., Chandra N., Haorah J. (2019). Animal models of traumatic brain injury and assessment of injury severity. *Molecular Neurobiology*.

[9] Pitotti C., David J. (2020). An evidence-based approach to nonoperative management of traumatic hemorrhagic shock in the emergency department. *Emergency Medicine Practice*.

[10] Kim S. H., Song S., Cho H. S., Park C. Y. (2019). Hybrid approach for treatment of multiple traumatic injuries of the heart, aorta, and abdominal organs. *Korean Journal Thoracic Cardiovascular Surgery*.

[11] Denil M. (2022). Manage unscheduled care in a multidisciplinary team on the basis of cooperation protocols. *Revue de l’infirmiere*.

[12] Wei F., Li Y. (2020). Successful management requiring multidisciplinary cooperation between seven departments for a large right-sided incarcerated traumatic diaphragmatic hernia: a case report and review of literature. *AME Case Rep*.

[13] Qian Z., Wang M., Xu T. (2022). Application of emergency specialist nursing combined with green channel mode in patients with limb amputation. *Applied Bionics and Biomechanics*.

[14] Zhang H., Zhang B., Chen J. (2021). The application of the emergency green channel integrated management strategy in intravenous thrombolytic therapy for AIS. *American Journal of Translation Resarch*.

[15] Larsson M., Forsman P., Hedenqvist P. (2017). Extracorporeal membrane oxygenation improves coagulopathy in an experimental traumatic hemorrhagic model. *European Journal of Trauma and Emergency Surgery*.

[16] Kim S. M., Kim S. I., Yu G. (2021). Role of thromboelastography in the evaluation of septic shock patients with normal prothrombin time and activated partial thromboplastin time. *Scientific Reports*.

[17] Crombie N., Doughty H. A., Bishop J. R. B. (2022). Resuscitation with blood products in patients with trauma-related haemorrhagic shock receiving prehospital care (RePHILL): a multicentre, open-label, randomised, controlled, phase 3 trial. *The Lancet Haematology*.

[18] Moore E. E., Moore H. B., Kornblith L. Z. (2021). Trauma-induced coagulopathy. *Nature Reviews Disease Primers*.

